# A multicenter phase II trial of neoadjuvant letrozole plus low‐dose cyclophosphamide in postmenopausal patients with estrogen receptor‐positive breast cancer (JBCRG‐07): therapeutic efficacy and clinical implications of circulating endothelial cells

**DOI:** 10.1002/cam4.1516

**Published:** 2018-05-07

**Authors:** Takayuki Ueno, Norikazu Masuda, Shunji Kamigaki, Takashi Morimoto, Futoshi Akiyama, Masafumi Kurosumi, Hitoshi Tsuda, Yoshiki Mikami, Sunao Tanaka, Satoshi Morita, Masakazu Toi

**Affiliations:** ^1^ Breast Surgical Oncology Breast Oncology Center Cancer Institute Hospital Japanese Foundation for Cancer Research Tokyo Japan; ^2^ Department of Breast Surgery School of Medicine Kyorin University Tokyo Japan; ^3^ National Hospital Organization, Osaka National Hospital Osaka Japan; ^4^ Sakai Municipal Hospital Osaka Japan; ^5^ Yao Municipal Hospital Osaka Japan; ^6^ Department of Pathology The Cancer Institute of Japanese Foundation for Cancer Research Tokyo Japan; ^7^ Department of Pathology Saitama Cancer Center Saitama Japan; ^8^ Department of Basic Pathology National Defense Medical College Saitama Japan; ^9^ Department of Diagnostic Pathology Kumamoto University Hospital Kumamoto Japan; ^10^ Department of Breast Surgery Graduate School of Medicine and Faculty of Medicine Kyoto University Kyoto Japan; ^11^ Department of Biomedical Statistics and Bioinformatics Graduate School of Medicine and Faculty of Medicine Kyoto University Kyoto Japan

**Keywords:** Breast cancer, chemo‐endocrine therapy, circulating endothelial cell, metronomic therapy, neoadjuvant

## Abstract

Neoadjuvant endocrine therapy has been reported to decrease tumor size, which leads to increased breast conservation rates. To improve the clinical response, metronomic chemotherapy with endocrine therapy is a promising strategy. A multicenter phase II single‐arm neoadjuvant trial with letrozole and cyclophosphamide was conducted. Eligibility criteria included postmenopausal status, T2–4 N0–1, and estrogen receptor‐positive breast carcinoma. Letrozole (2.5 mg) plus cyclophosphamide (50 mg) was given orally once a day for 24 weeks. The primary endpoint was the clinical response rate (CRR). To investigate anti‐angiogenic effects, circulating endothelial cells (CECs) were quantified using the CellSearch system. From October 2007 to March 2010, 41 patients were enrolled. The CRR was 67.5% (52.0–80.0%), which was above the prespecified threshold (65%). The conversion rate from total mastectomy to breast‐conserving surgery was 64% (18/28). Grade 3 or greater nonhematological toxicity was not reported. Clinical response was associated with improved disease‐free survival (DFS) (*P* = 0.020). The increase in CEC counts at 8 weeks was observed in nonresponders (*P* = 0.004) but not in responders. Patients with higher CEC counts at baseline or post‐treatment showed worse DFS than those with lower counts (*P* < 0.001 at baseline and = 0.014 post‐treatment). Multivariate analysis showed that post‐treatment CEC counts but not pretreatment counts were independently correlated with DFS (*P* = 0.046). In conclusion, neoadjuvant letrozole plus cyclophosphamide showed a good clinical response for postmenopausal patients with estrogen receptor‐positive breast cancer. CEC quantification is a promising tool for treatment monitoring and prognostic stratification for metronomic therapy following validation of our results in larger studies. Clinical trial registration number: UMIN000001331 Phase II study of neoadjuvant letrozole combined with low‐dose metronomic cyclophosphamide for postmenopausal women with endocrine‐responsive breast cancer (JBCRG‐07)

## Introduction

Neoadjuvant endocrine therapy (NET) is one of the treatment options for postmenopausal patients with endocrine‐responsive breast cancer. NET has been reported to result in decreased tumor size and increased breast conservation rates 1, 2, 3, 4, 5, 6. Because endocrine therapy is associated with lower toxicity than chemotherapy, NET is preferable to neoadjuvant chemotherapy, especially in older patients and those with worsening performance status. In order to further improve surgical outcome, it is important to increase the NET response rate without increasing adverse effects. Chemo‐endocrine therapy using metronomic chemotherapy is potentially useful in this regard.

Metronomic chemotherapy is the delivery of low doses of cytotoxic drugs at regular frequent intervals to avoid toxic side effects 7, 8. It has been suggested to act via multiple mechanisms in exerting anticancer effects, including anti‐angiogenesis, antitumor immune response, and direct anticancer action 9. Oral cyclophosphamide is one of the most commonly used metronomic agents and is administered alone or together with other drugs such as capecitabine and methotrexate 10, 11, 12, 13. Because metronomic chemotherapy shows anticancer effects via different mechanisms of action without overt toxic side effects, it is a good candidate in combination with endocrine therapy.

The combined administration of the aromatase inhibitor letrozole with low‐dose metronomic cyclophosphamide in elderly patients has been reported earlier 14. This randomized phase II trial showed an overall response rate (ORR) of 87.7% in patients assigned to receive letrozole plus cyclophosphamide, while letrozole alone showed an ORR of 71.9%. In addition, post‐treatment expression of Ki‐67 was significantly lower in tumors treated with the combined therapy than in tumors treated with letrozole alone. Thus, the combination of letrozole and oral cyclophosphamide appears effective and promising as neoadjuvant therapy.

We conducted a multicenter phase II single‐arm trial of neoadjuvant metronomic chemo‐endocrine therapy with letrozole and oral cyclophosphamide in Japan (Japan Breast Cancer Research Group‐07 trial: UMIN000001331). To investigate the possible role of anti‐angiogenic effects in metronomic chemo‐endocrine therapy, circulating endothelial cells (CECs) were quantified prior to and during the neoadjuvant treatment, and their association with treatment response and prognosis was examined.

## Patients and Methods

### Patients

Women with previously untreated, clinical T2–4 N0–1 and estrogen receptor (ER)‐positive breast carcinoma were enrolled in this study. Other inclusion criteria were (1) postmenopausal status and age 60 years or older; (2) 0–1 Eastern Cooperative Oncology Group performance status; and (3) written informed consent for participation in this study. Patients receiving agents that affect sex hormone status, such as hormone replacement therapy and raloxifene, were excluded. Consecutive patients who met the inclusion criteria and agreed to participate in the study were recruited from October 2007 to March 2010. Written informed consent was obtained from all patients who participated in the study. The study conforms to the provisions of the Declaration of Helsinki.

### Treatment

Patients received letrozole (2.5 mg) plus cyclophosphamide (50 mg) orally once a day for 24 weeks, and surgical therapy was conducted 1–4 weeks after the last administration of letrozole and cyclophosphamide. Anticipated surgery type before treatment and surgery type actually performed were compared to investigate whether preoperative therapy resulted in a higher breast conservation rate. Adverse events (AEs) were assessed in accordance with Common Terminology Criteria for Adverse Events (CTCAE) version 3.0.

No letrozole reduction was planned. Letrozole was planned to be interrupted when severe AEs occurred. Cyclophosphamide administration was delayed if the leukocyte count was <2000/mm^3^ or if the neutrophil count was <1000/mm^3^. In the event of grade 2 or greater cystitis and other grade 3 nonhematological AEs, cyclophosphamide was interrupted and postponed until recovery.

Postoperative radiation therapy, chemotherapy, trastuzumab, and endocrine therapy were given as per institutional practice.

The protocol was approved by the ethics committee in each institute.

### Endpoints

The primary endpoint was the clinical response rate, assessed using calipers, ultrasound (US), or computed tomography (CT)/magnetic resonance imaging (MRI) during the 24‐week neoadjuvant treatment period in the intention‐to‐treat (ITT) population. Tumor response was evaluated in accordance with RECIST ver. 1.0 15. Secondary endpoints included pathological therapeutic effects, breast conservation rate, safety assessed using CTCAE ver. 3.0, disease‐free survival (DFS), and overall survival (OS).

The target number of patients in the protocol was set at 40 based on the response rate of 88% in a previous report 14. On the assumption that the expected response rate was 85%, 33 patients would be required for verification of effectiveness under conditions of 65% threshold (based on NET results using letrozole alone), 5% one‐sided significance level, and 80% detection power.

### Pathological analyses

Pathological analyses were performed in a central laboratory. Tumor biopsy specimens before preoperative therapy were assessed for estrogen receptor, progesterone receptor (PgR), and human epidermal growth factor receptor type 2 (HER2). ER and PgR status were defined as positive for tumors with 10% or more positive tumor cells. HER2 positivity was determined as strong expression (3+) using immunohistochemistry or as HER2:CEP17 ratio >2.2 using fluorescence in situ hybridization 16. The pathological response was assessed using surgical samples following preoperative therapy. A pathological complete response (pCR) was defined as no residual invasive tumor cells in the mammary gland and lymph nodes. Grade 2 response was defined as reduction in tumor cells by more than two‐thirds (66%), and grade 1 was defined as reduction in tumor cells ≤ one‐third (33%). The Ki‐67 labeling index (LI) using the MIB1 antibody (Dako, Glostrup, Denmark) was calculated by counting positively stained tumor cells per 1000 tumor cells in the hot spots.

### Circulating endothelial cells

Blood samples were drawn into CellSave tubes (Veridex, LLC, NJ) prior to, at 8 weeks after treatment initiation, and at completion of the neoadjuvant treatment. Samples were sent to the central laboratory at Kyoto University where they were processed within 72 h after blood sampling. All evaluations were performed without prior knowledge of the patients’ clinical status. The CellSearch system was used for endothelial cell detection, as described previously 17, 18, 19. In brief, magnetic separation was performed using anti‐CD146 ferrofluids, followed by labeling with the nuclear stain 4,6‐diamidino‐2‐phenylindole (DAPI), a phycoerythrin‐conjugated anti‐CD105 antibody, and an allophycocyanin‐conjugated anti‐CD45 antibody. An additional channel was used for an anti‐CD34 antibody conjugated to FITC (clone AC136, Miltenyi, Biotech GmbH, Germany). CECs were defined as CD146^+^CD105^+^CD45^−^DAPI^+^ cells in this study. As CD34 is another maker that is positive in circulating endothelial cells, anti‐CD34 antibody was added to the additional channel 20. A gray‐scale charge‐coupled camera device was used to scan the entire chamber surface, and each captured frame was then evaluated for objects that were potential CEC candidates using image analysis software.

### Statistical analysis

Baseline characteristics of patients were summarized as mean (range) for continuous variables and number (%) for categorical variables. The clinical/pathological response rate and the breast conservation rate were calculated at 95% confidence intervals (CIs). AEs during treatment were tabulated based on their CTCAE grades. OS and DFS during follow‐up were estimated and compared using the Kaplan–Meier method and log‐rank test between groups stratified based on patient characteristics and clinical/pathological outcomes of the neoadjuvant treatment. In biomarker analysis, association of CECs (as continuous variables) with clinical response was evaluated using univariate logistic regression models. The optimal cut‐off value for each statistically significant biomarker to predict clinical response was determined using the Youden's index of the receiver operating characteristics (ROC) curve. Patients were stratified based on the cut‐off value into two groups, and the survival rate was compared between them. Multivariate survival analyses were performed using Cox proportional hazards models consisting of statistically significant variables from the survival analyses mentioned above. Multicollinearity was assessed using Spearman's rank correlation coefficient. To address data sparseness, Firth's penalized likelihood approach was applied in the regression analyses. A two‐sided *P*‐value below 0.05 was considered significant. Statistical analyses were performed using IBM SPSS Statistics 23.0 (IBM Corp., Armonk, NY) and R ver. 3.2.2 (R core team, R Foundation for Statistical Computing, Vienna, Austria).

## Results

### Population

From October 2007 to March 2010, 41 patients were enrolled in this study at four medical institutes in Japan (Fig. 1). One patient was excluded from the ITT population because of entry criteria violation (tumor size <2 cm). Six patients were further excluded from the per‐protocol set (PPS) due to entry criteria violation in three patients (higher transaminase in one, age less than 60 years in two patients), changing hospitals during the protocol treatment in one patient, and insufficient duration (<90%) of drug administration in two patients. Baseline characteristics of the entire population (safety population), the ITT population, and the PPS population are shown in Table 1.

**Figure 1:** CONSORT diagram of the study.

**Table 1:** Baseline characteristics of patients

Patient characteristics	Total enrolled (Safety population)	ITT	PPS
Number of patients	41	40	34
Age			
Ave. (range)	69.6 (57–82)	69.9 (57–82)	69.6 (61–80)
Staging			
T			
T1	1 (2.4)	0 (0.0)	0 (0.0)
T2	36 (87.8)	36 (90.0)	31 (91.2)
T3	4 (9.8)	4 (10.0)	3 (8.8)
N			
N0	36 (87.8)	35 (87.5)	29 (85.3)
N1	5 (12.2)	5 (12.5)	5 (14.7)
Receptor status			
ER			
+	41 (100.0)	40 (100.0)	34 (100.0)
−	0 (0.0)	0 (0.0)	0 (0.0)
PgR			
+	27 (65.9)	26 (65.0)	20 (58.8)
−	14 (34.1)	14 (35.0)	14 (41.2)
HER2			
+	9 (22.0)	9 (22.5)	5 (14.7)
−	32 (78.0)	31 (77.5)	29 (85.3)
Histological grade			
1	13 (31.7)	13 (32.5)	9 (26.5)
2	26 (63.4)	25 (62.5)	24 (70.6)
3	0 (0.0)	0 (0.0)	0 (0.0)
NA	2 (4.9)	2 (5.0)	1 (2.9)
			(): %

ER, estrogen receptor; ITT, intention‐to‐treat; PPS, per‐protocol set.

### Clinical and pathological response

The clinical response rate in the ITT population was 67.5% (52.0–80.0%), which was above the prespecified threshold (65%). Associations between clinical response and baseline characteristics were assessed. No baseline characteristics including Ki‐67 LI were associated with clinical response. Response rates in the HER2‐negative and HER2‐positive subgroups were 60% and 80%, respectively, which showed no statistically significant difference.

No patients achieved pCR. Seven patients (17.5%) showed grade 2 pathological responses and 28 (70%) showed grade 1 responses.

Changes in Ki‐67 LI were assessed based on clinical responses (Fig. 2). Ki‐67 LI decreased after treatment in both responders and nonresponders, and no difference in the decrease was observed based on clinical response.

**Figure 2:** Change in Ki67 labeling index according to clinical response. Ki67 labeling index decreased after the treatment in both responders and nonresponders (*P* < 0.001 for both). Representative images with Ki67 staining are shown (scale bar: 50 *μ*m).

### Surgical outcome

Among patients in the ITT population, breast‐conserving surgery was performed in 30 patients, and the breast‐conserving rate was 75% (30/40). Before treatment, breast‐conserving surgery and total mastectomy were anticipated in 12 and 28 patients, respectively. Eighteen patients who were anticipated to receive mastectomy before neoadjuvant treatment received breast‐conserving surgery. The conversion rate from total mastectomy to conserving surgery was 64% (18/28).

### Safety

Adverse events occurring in all enrolled patients are shown in Table 2. Twenty‐two patients (54%) had leukocytopenia, but most (17/22) of them were grade 1. Grade 3 leukocytopenia was observed in one patient. The most common nonhematological AE was arthralgia, which was observed in six patients. One patient was diagnosed with liver cancer 3 months after initiation of the neoadjuvant treatment, and the causal relationship with treatment is unlikely. No grade 3 or greater nonhematological toxicity was reported. No patients discontinued the treatment due to AE.

**Table 2:** Adverse events

Adverse event	All grade	Grade≧3
Diarrhea	1	0
Dry mouth/salivary gland	1	0
Stomatitis	1	0
Infection (cold sore)	1	0
Periodontal disease	1	0
Epigastric distress	1	0
Nausea	1	0
Anorexia	3	0
Liver cancer	1	0
Cystitis	2	0
Osteoporosis	2	0
Joint function:hand and finger joint stiffness	2	0
Pain⋅arthralgia	6	0
Pain⋅myalgia	1	0
Pain⋅headache	1	0
Perspiration	3	0
Postmenopausal syndrome (headache, dizziness)	3	0
Dizziness	1	0
Leukocytopenia	22	1
Thrombocytopenia	5	0
Anemia	7	0
Number of patients: 41		

### Survival analysis

Survival analyses were performed in the PPS. Among 34 patients, postoperative chemotherapy was given to seven patients. The median follow‐up period was 68.5 months (range: 18.1–86.5).

DFS at 5 years was 90.9% (95% CI: 48.4–90.4%). Three patients relapsed during follow‐up, one with axillary lymph node recurrence, one with chest wall recurrence, and one with lung metastasis. Overall survival at 5 years was 93.9% (95% CI: 74.4–97.0%). Two patients died during follow‐up, one with liver cancer and the other with myocardial infarction 3 years after treatment initiation. Baseline factors including T stage, nodal involvement, HER2 status, and types of surgery were not associated with DFS.

Associations of survival with clinical response and AEs were evaluated. Clinical response with US was associated with prognosis; responders showed better DFS than nonresponders (*P* = 0.020) (Fig. 3). Interestingly, leukocytopenia was associated with prognosis; patients with no or mild leukocytopenia (G0 or 1) had better DFS than those with severe leukocytopenia (G2 or 3) (*P* = 0.003) (Fig. 3). No other factors including pre‐ and post‐treatment Ki‐67 LI, changes in Ki‐67 LI, or HER2 status were associated with DFS or OS.

**Figure 3:** Disease‐free survival according to clinical response and leukocytopenia. Better clinical response and milder leukocytopenia were associated with a better disease‐free survival (*P* = 0.020 and 0.003, respectively).

### Circulating endothelial cells

Circulating endothelial cells were quantified prior to and during the neoadjuvant therapy. Their association with clinical response with US and prognosis were evaluated.

In nonresponders, CEC counts were significantly increased at 8 weeks (*P* = 0.004) compared with pretreatment counts, while in responders, no such increases were observed (*P* = 0.35) (Fig. 4). Similarly, CD34‐positive CEC counts were increased at 8 weeks in nonresponders (*P* = 0.003) but not in responders (*P* = 0.39). Baseline counts of CEC and CD34‐positive CEC did not correlate with treatment response.

**Figure 4:** Change in circulating endothelial cell count and clinical response. Nonresponders showed an increase in circulating endothelial cell count at 8 weeks (*P* = 0.004), while responders did not (*P* = 0.35).

The association between CEC counts and prognosis was evaluated. Cut‐off values for CEC and CD34‐positive CEC were determined using the Youden's index of ROC curves. Baseline counts of CEC and CD34‐positive CEC were significantly associated with DFS, and patients with higher counts of CEC and CD34‐positive CEC showed worse prognosis than those with lower counts (*P* < 0.001 and *P* = 0.004, respectively) (Fig. 5A). In addition, post‐treatment counts of CEC and CD34‐positive CEC were also significantly correlated with DFS (*P* = 0.014 and *P* = 0.008, respectively) (Fig. 5B).

**Figure 5:** (A) Disease‐free survival according to pretreatment CEC and CD34‐positive CEC count. Higher counts of CEC and CD34‐positive CEC showed a worse prognosis than lower counts (*P* < 0.001 and = 0.004, respectively). (B) Disease‐free survival according to post‐treatment CEC and CD34‐positive CEC count. Higher counts of post‐treatment CEC and CD34‐positive CEC showed a worse prognosis (*P* = 0.014 and 0.008, respectively).

Because clinical response and leukocytopenia were also associated with DFS, multivariate analyses of DFS, including clinical response, leukocytopenia, and pre‐ and post‐treatment counts of CEC, were performed. Interestingly, post‐treatment counts of CEC, but not pretreatment counts, were independently correlated with DFS (*P* = 0.046) (Table 3). A similar result was observed for CD34‐positive CEC (*P* = 0.043) (Table 3).

**Table 3:** Multivariate analysis of DFS

	Coef	SE (coef)	HR	Lower	Upper	*P*
CEC						
Response	−5.831	3.343	0.003	0	0.336	**0.007**
Leukocytopenia	1.909	1.317	6.745	0.748	212	0.087
CEC_pre	0.007	0.007	1.007	0.993	1.02	0.312
CEC_post	0.008	0.005	1.008	1.0001	1.021	**0.046**
CD34‐positive CEC						
Response	−6.143	3.429	0.002	0	0.298	**0.006**
Leukocytopenia	2.556	1.604	12.885	1.225	2668	**0.033**
CD34‐positive CEC_pre	0.008	0.007	1.008	0.995	1.022	0.201
CD34‐positive CEC_post	0.012	0.007	1.012	1.0004	1.03	**0.043**

CEC, circulating endothelial cell; DFS, disease‐free survival.

Bold means statistically significant.

## Discussion

In this study, we demonstrated that neoadjuvant metronomic chemo‐endocrine therapy with letrozole and cyclophosphamide showed a good response in Japanese postmenopausal women with ER‐positive breast cancer, with a conversion rate from mastectomy to breast‐conserving surgery of 64% and tolerable toxicity. In addition, increases in CEC counts at week 8 indicated poor response, and post‐treatment CEC counts showed a good and independent prognostic value.

One of the advantages of neoadjuvant treatment is an increase in breast‐conserving rate. The IMPAKT trial, which compared anastrozole, tamoxifen, and both in combination in the neoadjuvant setting, showed that the conversion rates from mastectomy to breast‐conserving surgery were 44%, 31%, and 24%, respectively 6. Thus, the conversion rate achieved in this study (64%) was higher than the rate in any endocrine treatment group of the IMPAKT trial. Another neoadjuvant endocrine study, the PROACT trial, compared anastrozole and tamoxifen 1. Although the conversion rate was not reported, the improvement in surgery including the conversion from mastectomy to breast‐conserving surgery was observed in 38.1% and 29.9% of the patients who received anastrozole and tamoxifen, respectively. Altogether, these results suggest that the combination of letrozole and cyclophosphamide would give a higher conversion rate than endocrine therapy alone.

In nonresponders, CEC counts increased at week 8, while in responders, such an increase was not observed. In our previous study, we showed that CEC counts done with the CellSearch system increased during neoadjuvant chemotherapy, especially during therapy involving taxane‐based regimens 17. Such increases have been suggested to contribute to angiogenesis and neovascularization in order to repair damaged tissues, including normal and cancerous tissues 21, 22, 23. Metronomic chemotherapy is expected to prevent such a vascular rebound in neovascularization, especially in tumor tissues, which is one of the suggested mechanisms for its anticancer effect. Therefore, it is conceivable that prevention of neovascularization due to metronomic chemotherapy led to maintained CEC counts in responders, while failure of such prevention resulted in increased CEC counts in nonresponders.

In our study, although CEC counts at both baseline and post‐treatment showed prognostic value, only post‐treatment CEC counts had independent prognostic power. Poor prognosis in patients with high post‐treatment CEC counts may be a result of insufficient anti‐angiogenic response with metronomic chemo‐endocrine therapy. This result seems consistent with the prognostic value of post‐treatment Ki‐67 LI in NET, which showed better prognostic power than pretreatment Ki‐67 LI 24, 25, 26, 27. Our results along with other reports suggest that biological responses, such as the antiproliferative response indicated by Ki‐67 LI and anti‐angiogenic response indicated by CEC counts after metronomic therapy, show more precise prognostic value than the baseline biology of tumors.

Leukocytopenia was associated with prognosis in this study. Severe leukocytopenia (G2 or G3) was associated with worse DFS. This seems contradictory to results reported with conventional chemotherapy in adjuvant settings for early‐stage breast cancer 28, 29, 30. These previous studies indicated that severe myelosuppression was associated with better prognosis in patients with breast cancer receiving CMF (cyclophosphamide, methotrexate, and 5‐fluorouracil) or CAF (cyclophosphamide, doxorubicin, and 5‐fluorouracil), suggesting that hematological toxicity due to conventional chemotherapy may represent biological activity of the drugs, resulting in improved prognosis. However, metronomic chemotherapy has been suggested to exert anticancer effects via different mechanisms of action compared to conventional chemotherapy, one of which is activation of antitumor immune response. Indeed, low‐dose cyclophosphamide has been implicated in activation of innate immunity 31, 32, 33. Therefore, myelosuppression during metronomic treatment may lead to insufficient immune activation, which might result in poor treatment efficacy in patients with severe leukocytopenia.

Although the objective response rate (67.5%) in our study appears a little lower than that (87.7%) in a previous report by Bottini et al. 14, some differences exist between the two studies. Bottini's study included only elderly patients, and thus, median patient age in our study was lower in comparison. More than half of the patients in Bottini's study had histological grade 3 tumors, while none of the patients in our study had grade 3 tumors. The clinical response was assessed using calipers in Bottini's study, while it was assessed with calipers, US, and CT/MRI in our study. These differences might have contributed to different response rates in the two studies.

This study was limited in terms of some parameters. One of its biggest limitations was its small sample size. Because this was a phase II trial investigating clinical efficacy and tolerability of combined treatment with letrozole and low‐dose cyclophosphamide, the sample size was set at 40. In order to validate the clinical utility of the treatment, a larger study is warranted. It is also important to interpret the results including the prognostic analysis with this sample size cautiously. To confirm the prognostic value of CEC, it is necessary to conduct a larger study in which CECs are serially measured. The definition of ER and PgR positivity is another issue. In 2010, the American Society of Clinical Oncology/College of American Pathologists recommended that ER and PgR assays be considered positive if there are at least 1% positive tumor nuclei in the sample on testing with appropriate controls 34. Because this study started in 2007, the old criteria of ER and PgR were used. Thus, future studies to validate our results should be conducted with the new definition of ER and PgR positivity. Another limitation was that this was a single‐arm study in which chemo‐endocrine therapy was not compared with either endocrine therapy alone or metronomic chemotherapy alone. It is, therefore, not clear whether combined administration of letrozole with metronomic cyclophosphamide resulted in a better outcome than letrozole or cyclophosphamide alone would have in this population. A randomized controlled study would be required for such a comparison in a larger confirmative study.

In conclusion, metronomic chemo‐endocrine therapy with letrozole plus cyclophosphamide showed a good response and was tolerated in Japanese postmenopausal patients with ER‐positive breast cancer. An increase in CEC counts during the treatment was associated with poor response, and post‐treatment CEC counts as well as clinical response were independent prognostic factors. The combination of letrozole and cyclophosphamide could be an option for postmenopausal women with ER‐positive breast cancer. CEC quantification would be a promising tool for treatment monitoring and prognostic stratification following validation of our results in larger prospective studies.

## Conflict of Interest

T Ueno has received honoraria from Chugai Pharmaceutical Co., Ltd., Eisai Co., Ltd., Novartis Pharma K.K. N Masuda has received honoraria from Chugai Pharmaceutical Co., Ltd., Astra Zeneca K.K. S Morita has received honoraria from Chugai Pharmaceutical Co., Ltd. M Toi has received research funding from Taiho Pharmaceutical Co., Ltd., Chugai Pharmaceutical Co., Ltd., Eisai Co., Ltd., Shimadzu Corporation, C & C, Japan Breast Cancer Research Group, Astra Zeneca K.K., AFI Technology, Daiichi‐Sankyo Co., Ltd.
